The article "Transplacental Transmission of Theileria equi Is Not a Common Cause of Abortions and Infection of Foals in Israel" was published in 2020. Journal: Animals (Basel).

# Transplacental Transmission of *Theileria equi* Is Not a Common Cause of Abortions and Infection of Foals in Israel

**DOI:** 10.3390/ani10020341

**Published:** 2020-02-21

**Authors:** Sharon Tirosh-Levy, Yuval Gottlieb, Lea Mimoun, Monica L. Mazuz, Amir Steinman

**Affiliations:** 1 Koret School of Veterinary Medicine, The Robert H. Smith Faculty of Agriculture, Food and Environment, The Hebrew University of Jerusalem, 7610001 Rehovot, Israel; sharontirosh@gmail.com (S.T.-L.); gottlieb.yuval@mail.huji.ac.il (Y.G.); lea.mimoun@mail.huji.ac.il (L.M.); 2 Division of Parasitology, Kimron Veterinary Institute, 50250 Bet Dagan, Israel; MonicaL@moag.gov.il

**Keywords:** abortion, equine, equine piroplasmosis, *Theileria equi*, transplacental-transmission

## Abstract

**Simple Summary:**

*Theileria equi* is a parasite of horses that is mainly transmitted by ticks but has also been reported to be transmitted from infected mares to their foals during pregnancy. This type of transmission may lead to abortion or to the birth of sick or infected foals. Little data are available regarding the magnitude of this type of transmission, although *T. equi* is considered to be a major cause of abortion in some areas. The aim of this study was to determine if *T. equi* is often transferred from mares to foals in an area where this parasite is abundant. We found that although the majority of aborting mares carried the parasite, none of the aborted fetuses were infected. Further, in a farm where all mares were infected, only one foal was infected by 6 months of age, and that infection was probably not from its dam. Although the number of inspected animals was small, our findings suggest that *T. equi* is not frequently transferred to foals during pregnancies of carrier mares.

**Abstract:**

Although the main route of transmission of *Theileria equi* is through tick feeding, transplacental transmission is also possible and may lead to abortion, or to the birth of a sick or carrier foal. The aim of this study was to evaluate the role of *T. equi* as a cause of abortions in Israel and the risk of foals being infected at a young age. Eight aborting mares were serologically evaluated for exposure to *T. equi* via the immunofluorescence antibody test (IFAT) and their aborted fetuses were evaluated using PCR and qPCR. In addition, five mares and their foals (aged 4–6 months) from a highly endemic farm were tested for *T. equi* infection using IFAT, PCR and qPCR. Five of the eight aborting mares were seropositive for *T. equi*; however, none of the aborted fetuses was infected. All five mares from the endemic farm were subclinically infected with *T. equi*. Of their five foals, one was infected, with relatively high parasitemia and different parasite genotype than its dam’s, suggesting another source of infection. The results of this study suggest that transplacental transmission of *T. equi* is not common and does not appear to be a prominent cause of abortion in chronically infected mares.

The article "Transplacental Transmission of Theileria equi Is Not a Common Cause of Abortions and Infection of Foals in Israel" was published in 2020. Journal: Animals (Basel).

## 1. Introduction

*Theileria equi* is a tick-borne hemoparasite of equids that is endemic in many parts of the world and poses an enzootic threat to currently non-endemic areas [1]. Clinical signs of disease are attributed mainly to hemolytic anemia caused by parasite replication in the host red blood cells. Disease may range from subclinical to life-threatening and infection usually results in life-long carriage of parasites [1,2].

The main route of infection of horses is through tick infection. The sporozoites present in the tick salivary glands are transmitted via saliva during the blood meal. Transplacental transmission of parasites has also been documented and may result in late-term abortion or neonatal piroplasmosis, which often lead to the death of the infected foal [3,4,5,6,7,8]. In some endemic areas, *T. equi* is a significant cause of abortion and has considerable economic consequences due to fetal loss and foal deaths [9]. It has also been demonstrated that in some cases, transplacental transmission from subclinically infected mares may result in normal foaling and apparently healthy infected foals [10,11].

Foals of *T. equi* carrier mares receive anti-*T. equi* antibodies from the colostrum which persist up to four months [12,13]. In endemic areas, early exposure of foals to *T. equi* is probably important to induce enzootic stability and protective immunity, which lowers the risk of developing clinical signs of infection [1,10].

*T. equi* is endemic in Israel, with some hyper-endemic regions [14,15]. Thus, clinical cases are infrequently reported in horses resident in these regions. Cases of neonatal piroplasmosis are occasionally reported [6]; however, *T. equi* is not routinely checked in cases of abortion. The aim of this study was to evaluate the role of *T. equi* as a causative agent of abortions and the chance of foals being infected at a young age in an endemic area, such as Israel.

## 2. Materials and Methods 

### 2.1. Sample Collection 

Aborted fetuses and placentas were collected as a part of a surveillance study of equine abortions, along with sera of the aborting mares by their attending veterinary practitioners. The fetuses and placentas were dissected and kept at 4 °C until DNA extraction.

Foals’ and mares’ blood was collected as a part of another long-term surveillance study in a farm of 30 horses reared on pasture in the Golan Heights. The farm was sampled on several occasions during 2014–2017, and in August 2017, five of the mares had foals aged 4–6 months. The reason for targeting this age group was to examine foals after the elimination of maternal antibodies, to ensure that the serological results represent exposure of the foal and not of its dam.

The article "Transplacental Transmission of Theileria equi Is Not a Common Cause of Abortions and Infection of Foals in Israel" was published in 2020. Journal: Animals (Basel).

Blood was collected from the jugular vein of all mares and foals and placed in sterile vacuum tubes containing ethylenediamine tetraacetic acid (EDTA) and tubes without an anticoagulant. Sera were obtained from the clotted blood samples by centrifugation (4000G for 10 min). Whole blood and serum samples were kept at −20 °C until processing.

Sample collection was performed under the horse owners’ consent, and the study was approved by the Internal Research Committee of the Koret School of Veterinary Medicine–Veterinary Teaching Hospital (KSVM-VTH/23_2014, KSVM-VTH/02_2018).

### 2.2. Serological Screening

Serological screening for the presence of anti-*T. equi* antibodies was performed on sera from all aborting mares, on the chest fluid of most aborted fetuses (when available), and on sera from the mares and foals from the endemic farm, using immunofluorescence antibody test (IFAT).

Antigen was prepared in-house from *T. equi*-infected erythrocytes from culture and stored in −80 °C until use. Slides were dried at 37 °C for 30 min and fixed in acetone for 10 min and air-dried before use. Sera were diluted to 1:80 with bovine serum albumin (BSA) as a cut-off value for screening. A volume of 35 µL of serum was added to each antigen-containing well and incubated in a humid chamber at 37 °C for 30 min. Slides were washed for 10 min in Phosphate buffer solution (PBS) before application of 35 µL anti-horse antigen diluted 1:120 with BSA, and incubation at 37 °C for 30 min in a humid chamber. Slides were later washed for 10 min in PBS, dried, mounted with glycerol/PBS 1:1 and inspected under a fluorescence microscope. Positive and negative control samples were added to each run.

### 2.3. DNA Extraction

DNA was extracted from 50 µL of whole blood from each sample, diluted in 350 µL double distilled water (DDW) using a commercial kit (RTP Pathogen Kit, Stratec, Germany), according to the manufacturer’s instructions (mare samples from 2015); or from 100 µL of whole blood using a commercial kit (DNeast blood and tissue kit, QIAGEN, Hilden, Germany), in accordance with the manufacturer’s instructions (mares’ and foals’ samples from 2017). DNA from fetal tissues and placentas was extracted using the Maxwell^®^ RSC instrument and extraction kit (Promega, Wisconsin, USA).

### 2.4. Polymerase Chain Reaction (PCR) for the Detection of T. equi 

A 400 bp segment of the *T. equi* 18S r RNA gene was amplified by PCR using the primers *Bec-UF2* (TCGAAGACGATCAGATACCGTCG) and *Equi-R* (TGCCTTAAACTTCCTTGCGAT), as previously described [16,17]. The reaction was repeated for the mare and foal samples from 2017 as nested PCR using the external primers *NBabesia1F* (AAGCCATGCATGTCTAAGTATAAGCTTTT) and *18SRev-TB* (GAATAATTCACCGGATCACTCG), as previously described [15], and the internal primers as above, using 2 µL of the original reaction as a template.

The article "Transplacental Transmission of Theileria equi Is Not a Common Cause of Abortions and Infection of Foals in Israel" was published in 2020. Journal: Animals (Basel).

All positive PCR products were cleaned using Exonuclease I and Shrimp alkaline phosphatase (New England Biolabs Inc., Massachusetts, US) and sent for sequencing (Macrogen Europe, Amsterdam, The Netherlands). Sequences were inspected and trimmed using Chromas software version 2.6 (Technelysium Pty Ltd., South Brisbane, Australia) and were confirmed as *T. equi* with over 97% homology to *T. equi* MK063842 (genotype A) or MK392059 (Genotype D) GenBank references using the BLAST algorithm (http://www.ncbi.nlm.nih.gov/BLAST, last accessed September 2019).

### 2.5. Quantification of T. equi Parasitemia Using Quantitative Real-Time PCR Reaction (qPCR)

Parasitemia levels in the aborted fetuses and in the mares and foals from the endemic farm were assessed using qPCR with TaqMan minor groove binder (MGBTM) probe targeting *T. equi* equine merozoite protein-1 (ema-1) gene [18]. Samples were tested in duplicate and were considered positive when both duplicates were positive. A clean PCR product was used to prepare the standard curve, and gene copy number (gcn) was calculated from the molecular weight and gene length: gcn = (ng × gcn/mole)/(bp × ng/g × g/mole of bp). A standard curve of 1–10^7^ copies was used to determine the copy number in each sample. The cut-off for parasite detection was set at 1 copy. A second standard curve was prepared using DNA extracted from serial dilutions of *T. equi* blood culture with known parasitemia (% parasitized erythrocytes (PE)), and parasitemia levels was calculated from gene copy number using transformation between the two curves.

## 3. Results

### 3.1. T. equi in Mares and Aborted Fetuses

Eighteen serum samples were collected from aborting mares, thoracic fluid was available from fifteen aborted fetuses, and DNA was extracted from placentas (five cases), fetal livers (four cases) and fetal spleens (three cases). From four fetuses, more than one DNA sample was obtained (liver and spleen in two cases, liver and placenta in the other two cases).

Fifteen of the mares were Arabians, one Warmblood, one Singlefoot and one Quarter horse. Their ages ranged between 4 and 22 years (mean = 10.9, SDV = 5.4). All mares were housed in stalls, and half of them had access to paddocks or pasture. Sixteen mares had previous pregnancies with normal foals, the other two mares were primiparous.

The article "Transplacental Transmission of Theileria equi Is Not a Common Cause of Abortions and Infection of Foals in Israel" was published in 2020. Journal: Animals (Basel).

Eleven of the aborting mares and none of the fetuses were seropositive for *T. equi*. *T. equi* DNA was not found in any of the aborted fetuses tested by both PCR and qPCR.

### 3.2. T. equi in Mares and Foals

Five paired mares and foals were sampled in August 2017 in a *T. equi* highly-endemic farm. The farm was a part of a surveillance study during 2015, and all five mares had also been sampled then. All five mares were mixed-breed horses aged 6–16 years in 2017 (mean = 9.4, SDV = 3.9) and were turned out to pasture. All mares were found to be infested with ticks during both samplings (Table 1). The foals were 4–6 months old and comprised three fillies and two colts. Ticks were present on all foals during sampling (Table 1).

All five mares were positive for *T. equi* at both time points in all detection methods (IFAT, PCR and qPCR). All parasites from 2017 were classified as *T. equi* 18S rRNA genotype D, while in 2015, three samples were classified as genotype D and the other two as genotype A. Parasite loads in all mares were low (mean = 6.48, SDV = 2.98 gcn in 2015 and mean = 1.99, SDV = 0.98 gcn in 2017), corresponding with parasitemia levels of 5.9 × 10^−5^–1.9 × 10^−4^% PE (Table 1).

Only one of the five foals was positive for *T. equi*, using all detection methods, with a considerably high parasite load (1416.89 gcn, 0.075% PE and was classified as genotype A (Table 1).

## 4. Discussion

Although *T. equi* is highly endemic to Israel, it does not appear to be a major cause for abortion, and transplacental transmission does not appear to occur often. Abortions as a result of *T. equi* infection or carriage, as well as neonatal piroplasmosis (both clinical and subclinical) are stated to be common [4]; however, few studies were conducted to support this claim. Most of the literature describes clinical case reports with fatal consequences [3,5,6,8]. Few cases described transplacental transmission that resulted in healthy foals. A study from the UK identified four positive foals that were born in a non-endemic area, with no potential exposure to ticks, to imported carrier dams and sires [11]. A study in Trinidad surveyed 111 pregnant mares of which 27 tested positive for *T. equi* by PCR. Although it also described 19.8% abortions and four *T. equi*-positive healthy foals, the cause of abortions was not tested, nor was the percentage of abortions in the *T. equi* positive mares [19,20]. In South Africa, which is an endemic region, *T. equi* was reported as the cause of 11% of equine abortions [9] and demonstrated that intrauterine transmission occurs as early as the second trimester and may result in the birth of subclinically infected foals [10]. In the current study, although eleven of the eighteen aborting mares and all five mares with normal foals were positive for *T. equi*, only one healthy foal tested positive, and in this case, post-natal infection could not be ruled out as the *T. equi* 18S rRNA genotype differed between the mare and the foal.

The article "Transplacental Transmission of Theileria equi Is Not a Common Cause of Abortions and Infection of Foals in Israel" was published in 2020. Journal: Animals (Basel).

Not all intrauterine infections result in clinically-infected foals or fetuses. Therefore, identification of parasites in aborted fetuses or sick foals does not necessarily imply that is the cause of abortion or disease. Most case reports of neonatal disease usually report considerably high parasitemia (40–60% PE) in the infected foals, which supports the assumption that *T. equi* is the cause of disease and fatality [3,5]. However, in cases of abortion or stillbirth, parasites were usually detected in fetal samples but were not quantified [8]. In this study, we aimed to detect and quantify parasite DNA in the placenta and fetal tissue, as well as to detect anti-*T. equi* antibody response in the fetuses. Since normal equine placenta is not permeable to antibody passage, detection of antibodies in the fetus suggests either exposure to the parasite or placental damage. However, neither parasite DNA nor specific antibodies were detected in any of 18 aborted fetuses.

It is possible that transplacental transmission can occur and lead to low rates of infection in the foals; thus, the foals are born apparently healthy carriers of *T. equi*. In this study, none of the five carrier mares transmitted *T. equi* to their offspring. Thus, it appears that transplacental transmission is not a significant way to spread the parasites from an epidemiological view. It is possible that the significance of this transmission is underestimated due to the limited number of cases, and a large-scale survey should be performed to thoroughly evaluate the role of transplacental transmission in the epidemiology of EP.

Parasitemia levels in subclinical carriers are usually low and have been documented to range between 1.99 and 1000 parasites per µL blood [21], equivalent to 2.2 × 10^−5^–0.011% PE. Quantification of parasitemia in the carrier mares in this study concurred with this range (5.9 × 10^−5^–1.9 × 10^−4^% PE). The infected foal, however, had considerably higher parasitemia (0.075% PE) and, although subclinical, may indicate novel infection, which is also supported by the finding that *T. equi* 18S rRNA genotype differed between the mare and the foal. We tested 4–6-month-old foals assuming that by this age maternal antibodies are eliminated [12,13] and anti-*T. equi* antibodies result from exposure to the parasite. The fact that in this study foals were serologically negative for *T. equi* may indicate that by this age, maternal antibodies have been, indeed, eliminated [12,13], and an encounter with the parasite is required to stimulate adaptive immune response.

The article "Transplacental Transmission of Theileria equi Is Not a Common Cause of Abortions and Infection of Foals in Israel" was published in 2020. Journal: Animals (Basel).

Molecular tools are used to characterize parasite strain and help to identify the source of infection. The 18S rRNA gene is commonly used in the characterization of piroplasms and other epicomplexan parasites [22,23]. In Israel, we found that *T. equi* 18S rRNA genotype D is more common in highly endemic farms, while genotype A is more associated with less endemic areas, with clinical cases and within the vector ticks (Sharon Tirosh-Levy, The Hebrew University of Jerusalem, unpublished results). Seventy-four per cent of the isolates identified in the farm where the mares and foals were sampled were of genotype D. The fact that two mares were classified as genotype A in 2015 and as D in 2017 may reflect re-infection, or a shift in the balance in co-infection with several strains. The only positive foal was infected with *T. equi* genotype A. This may support the hypothesis that this genotype is more often associated with susceptible animals and de novo infection. The infected foal may have been infected by the mare during pregnancy or by a tick after birth. The different genotype in the mare may support the latter assumption, and that colostral protection may had played a role in the absence of clinical disease [13], even if infected with a different parasite strain. The only other reports of transplacental transfer that had molecular classification of the infecting genotype were one case report from Israel [6] and five from Trinidad [5,19], and all were classified as genotype A. However, since all equine isolates from Trinidad were of the A genotype, little can be deduced as to the likelihood of a certain genotype being maternally transmitted.

## 5. Conclusions

Our results suggest that transplacental transmission may play a minor role in the epidemiology of equine Theileriosis in endemic areas. The carrier status of the mares may not imply the infection of the foal or a higher risk of abortion related to the presence of parasites.

## Figures and Tables

**Table 1:** *T. equi* carriage in mares (M1-5) and their foals (F1-5) from an endemic farm. The characteristics of each horse and the results of the serological and molecular tests are stated. The mares were sampled on two occasions, during 2015 and during 2017. F-female, M-male, IFAT-immunofluorescence antibody test, PCR-polymerase chain reaction for *T. equi* 18S rRNA gene, qPCR-TaqMan real time PCR for *T. equi ema-1* gene, qPCR results are stated as gene copy number, Genotype- *T. equi* genotype characterized according to a ~400 b sequence of its 18S rRNA gene.

Horse	Age	Breed	Sex	Housing	Sample 1	Ticks	IFAT	PCR	qPCR	Genotype	Sample 2	Ticks	IFAT	PCR	qPCR	Genotype
M1	9y	Mixed	F	Pasture	2015	+	+	+	8.14	D	2017	+	+	+	2.05	D
M2	6y	Mixed	F	Pasture	2015	+	+	+	10.02	D	2017	+	+	+	1.5	D
M3	16y	Mixed	F	Pasture	2015	+	+	+	4.29	D	2017	+	+	+	3.64	D
M4	9y	Mixed	F	Pasture	2015	+	+	+	2.634	A	2017	+	+	+	1.12	D
M5	7y	Mixed	F	Pasture	2015	+	+	+	7.33	A	2017	+	+	+	1.65	D
F1	4m	Mixed	M	Pasture							2017	+	-	-	0	-
F2	4m	Mixed	F	Pasture							2017	+	-	-	0	-
F3	4m	Mixed	F	Pasture							2017	+	+	+	1416.89	A
F4	6m	Mixed	F	Pasture							2017	+	-	-	0	-
F5	5m	Mixed	M	Pasture							2017	+	-	-	0	-
